The article "An amperometric H2O2 biosensor based on hemoglobin nanoparticles immobilized on to a gold electrode" was published in 2017. Journal: Biosci Rep.

# An amperometric H_2_O_2_ biosensor based on hemoglobin nanoparticles immobilized on to a gold electrode

**DOI:** 10.1042/BSR20170194

**Published:** 2017-07-17

**Authors:** Vinay Narwal, Neelam Yadav, Manisha Thakur, Chandra S. Pundir

**Affiliations:** 1 Department of Biochemistry, M.D. University, Rohtak, Haryana, India; 2 Centre for Biotechnology, M.D. University, Rohtak, Haryana, India; 3 Dr B.R. Sur Homeopathic Medical College and Hospital, Department of Pathology, New Delhi, India

**Keywords:** H2O2, Hemoglobin nanoparticles, Gold electrode, Serum, H2O2 biosensor

## Abstract

The nanoparticles (NPs) of hemoglobin (Hb) were prepared by desolvation method and characterized by transmission electron microscopy (TEM), UV spectroscopy and Fourier-transform IR (FTIR) spectroscopy. An amperometric H_2_O_2_ biosensor was constructed by immobilizing HbNPs covalently on to a polycrystalline Au electrode (AuE). HbNPs/AuE were characterized by scanning electron microscopy (SEM), cyclic voltammetry (CV) and electrochemical impedance spectra (EIS) before and after immobilization of HbNPs. The HbNPs/AuE showed optimum response within 2.5 s at pH 6.5 in 0.1 M sodium phosphate buffer (PB) containing 100 μM H_2_O_2_ at 30°C, when operated at –0.2 V against Ag/AgCl. The HbNPs/AuE exhibited *V*_max_ of 5.161 ± 0.1 μA cm^−2^ with apparent Michaelis-Menten constant (*K*_m_) of 0.1 ± 0.01 mM. The biosensor showed lower detection limit (1.0 μM), high sensitivity (129 ± 0.25 μA cm^−2^ mM^−1^) and wider linear range (1.0–1200 μM) for H_2_O_2_ as compared with earlier biosensors. The analytical recoveries of added H_2_O_2_ in serum (0.5 and 1.0 μM) were 97.77 and 98.01% respectively, within and between batch coefficients of variation (CV) were 3.16 and 3.36% respectively. There was a good correlation between sera H_2_O_2_ values obtained by standard enzymic colorimetric method and the present biosensor (correlation coefficient, *R^2^* =0.99). The biosensor measured H_2_O_2_ level in sera of apparently healthy subjects and persons suffering from diabetes type II. The HbNPs/AuE lost 10% of its initial activity after 90 days of regular use, when stored dry at 4°C.

## Introduction

Hydrogen peroxide (H_2_O_2_) is an incompletely reduced metabolite of oxygen that has a diverse array of physiological and pathological effects within living cells, depending on the extent, timing and location of its production. Characterization of the cellular functions of H_2_O_2_ requires measurement of its concentration selectively in the presence of other oxygen metabolites with spatial and temporal fidelity in live cells [1]. H_2_O_2_ is one of the reactive oxygen species (ROS) amongst others like superoxide anion (O_2_^•−^), hydroxyl radical (OH^•^), hydroxyl ion (OH^−^). The higher concentration of H_2_O_2_ is associated with diabetes, atherosclerosis, and ageing, as it generates free hydroxyl radicals, which cause oxidative damage to the tissue components such as lipids and proteins beside DNA [2,3]. For the measurement of H_2_O_2_ in biological fluids, several sensitive methods based on horseradish peroxidase (HRP) and artificial substrates (such as Amplex Red and 3,5,3′,5′-tetramethylbenzidine) or on ferrous oxidation in the presence of xylenol orange (FOX) have been developed [4]. The rapid and accurate determination of H_2_O_2_ is very important, as it is not only the product of the reactions catalyzed by many highly selective oxidases, but also employed in various fields such as food, pharmaceutical, biology, medicine, industry and environmental analysis [5]. Hyperglycemia is one of the major ways of inducing ROS and endothelial dysfunction in patients with diabetes [6]. The imbalance between the production of ROS and the endogenous antioxidant mechanism to counteract the effect of ROS or repair the resulting damages generate oxidative stress [7]. The determination of H_2_O_2_ in diabetics helps in evaluating their oxidative stress status. By maintaining a good diabetic control and implementing strategies including supplementation of antioxidant micronutrients (vitamins E and C, β-carotene) will reduce the oxidative stress and thus help in reducing the risk of chronic complications [8]. Several methods, such as titrimetry [5], spectrometry [9], chemiluminescence [10], fluorimetry [11], chromatography [12], and electrochemical techniques [13,14] have been reported for this purpose. Amongst these techniques, the electrochemical techniques are preferable, because of their simplicity, low cost, high sensitivity, rapidity, and selectivity. The proteins containing heme groups, such as hemoglobin (Hb), myoglobin, and cytochrome* c* possess peroxidase-like for reduction of H_2_O_2_, due to the electroactive center of heme [15-17]. Amongst these, Hb is more suitable for H_2_O_2_ biosensor, because of its known structure, commercial availability at low cost and is relatively more stable. Thus the biosensors using native Hb were more specific with reduced fabrication cost [18,19]. The native Hb has been immobilized on to various types of nanocomposites for construction of H_2_O_2_ biosensor such as Hb/Pluronic P123-nanographene platelet (NGP) [20], Hb/collagen microbelt [21], Hb/Ag sol films [22], Hb/AuNPs/L-Cysteine (L-cys)/*p*-aminobenzene sulphonic acid (*p*-ABSA)/Pt disk [24], Hb/collagen-multiwall carbon nanotubes (c-MWCNT) [24], DNA–Hb/Au [25]. The various supports used for the H_2_O_2_ biosensors are: platinum nanoparticles (NPs) (PtNPs)/reduced graphene oxide (RGO)/chitosan (CS)/ferrocene (Fc) [28], self-assembled dipeptide (DP)-gold NPs (AuNPs)/HRP/glassy carbon electrode (GCE) [29], graphene capsules (GRCAPS)/HRP/indium tin oxide (ITO) [30], HRP/poly(aniline-co-N-methyllanthionine) (PAN-PNMThH) [31], electrochemically reduced graphene oxide (ERGO)/GCE [32], 3,3′,5,5′-teramethylbencidine (TMB)/HRP/polydimethylsiloxane (PDMS)/tetraethylorthosilicate (TEOS)/silicon oxide NPs (SiO_2_NPs) [33], turnip tissue paper (TTP)/SPCE [34], GPtNPs [35], PtRu/3DGF [36], cytochrome *c* (Cytc)/nickel oxide nanaoparticles (NiONPs)/c-MWCNT/polyaniline (PANI)/Au [37]. However, these methods involve the complex strategies for construction of working electrode and have poor detection limit and narrow linear range. Hence, there is a need for development of an efficient and reliable analytical device that can provide high sensitivity, facile operation, and quick response to the H_2_O_2_ molecule. In recent years, protein NPs have been employed in the construction of improved biosensors due to their exceptional electronic, optical, mechanical, and thermal properties [26]. AuE offers many attractive features such as good conductor of electricity, low cost, low background current, and easy availability [27]. The present work describes the construction of an H_2_O_2_ biosensor based on covalent immobilization of HbNPs on to AuE, its characterization, evaluation, and application for amperometric determination of H_2_O_2_ in sera of diabetic patients.

The article "An amperometric H2O2 biosensor based on hemoglobin nanoparticles immobilized on to a gold electrode" was published in 2017. Journal: Biosci Rep.

## Experimental procedures

### Materials

Hb, Tris buffer, NAD^+^, D-Glucose, uric acid, urea, glucose, ascorbic acid, potassium chloride, silica gel from SRL, Mumbai; sulphuric acid from Qualigens Fine Chemicals, Mumbai were used. Au wire (diameter: 2 mm) for the preparation of AuE was purchased from a local jewellery shop. Sera samples of apparently healthy subjects and persons suffering from diabetes type II were collected from local PGIMS hospital. All other chemicals were of analytical reagent (AR) grade. Double distilled water (DW) was used throughout the experimental studies.

### Instruments used

Potentiostat/galvanostat (Make: Autolab, model: AUT83785, manufactured by Eco Chemie, The Netherlands) with a three electrode system consisting of Pt wire as an auxillary electrode, an Ag/AgCl electrode as a reference electrode and HbNPs immobilized on to polycrystalline Au as a working/enzyme electrode. SEM (Zeiss EV040, U.S.A.), UV spectrophotometer (make: Shimadzu, Japan, model: 1700), X-ray diffractometer (XRD) (make: 122 Rigaku, D/Max2550, Tokyo, Japan), Fourier transform IR (FTIR) spectrometer (Thermo Scientific, U.S.A.) were used.

The article "An amperometric H2O2 biosensor based on hemoglobin nanoparticles immobilized on to a gold electrode" was published in 2017. Journal: Biosci Rep.

### Preparation of HbNPs

The HbNPs were prepared by desolvation method. To the Hb solution (1 mg/ml), 5 ml of absolute ethanol was added dropwise at a rate of 0.1–0.2 ml/min under continuous stirring at a speed of 500 rpm. The desolvating agent encouraged the aggregation of protein molecules into small NPs by eliminating water molecules amongst them. In the same way, process was followed by addition of 1 ml of 1% glutaraldehyde solution into the reaction mixture. The mixture was kept under the similar stirring conditions at 4°C for 24 h to ensure complete cross-linking of HbNPs. Such a high concentration of glutaraldehyde is likely to provide intermolecular cross-linking of HbNPs molecules through Schiff’s base. Besides, above all the enzyme HbNPs thus formed were thiol functionalized by adding 0.02 g/ml cysteamine solution (0.02 g/ml) to HbNPs suspension under constant stirring for 5–6 h. Last, HbNPs were separated from the supernatant by centrifuging NPs suspension at 1200×***g*** for 10 min at 4°C, followed by redispersion of HbNPs in 0.1 M phosphate buffer (PB) (pH 7.3) and sonication for 5 min. Moreover, it is assumed that α-NH_2_ group of cysteamine reacts with excess unreacted –CHO groups of glutaraldehyde cross-linked Hb molecules to form Schiff’s base. Thus, the glutaraldehyde cross-linked HbNPs get functionalized with –SH groups. These –SH functionalized HbNPs were stored at 4°C until use [38].

### Characterization of HbNPs

HbNPs were characterized by recording their TEM images, UV and visible spectra and FTIR spectra. The size and shape of HbNPs were measured by a high-resolution transmission electron microscope, Zeiss EM 912, at an accelerating voltage of 120 kV. TEM samples of the HbNPs were prepared by placing the product solution on to the carbon-coated copper grids, allowing the solvent to evaporate in air. UV absorbance of HbNPs dispersed in 0.1 M sodium PB (pH:7.0) was recorded in the range from 200 to 600 nm at an interval of 50 nm, using UV spectrophotometer (make: Shimadzu, Japan, model 1700). FTIR spectra of the HbNPs were measured by FTIR spectrometer (Thermo Scientific, U.S.A.) using the standard KBr method over a range of 500–4000 cm^−1^.

### Preparation of HbNPs modified Au electrode

Thiol groups on the surface of HbNPs provide a facile way for attachment of HbNPs on the surface of Au electrode (AuE). Before immobilization, the cleaned bare AuE was scanned over the 0–0.5 V range in freshly prepared 0.2 M H_2_SO_4_ until the voltammogram characteristic of the clean polycrystalline Au was established. The polycrystalline AuE was placed in the HbNPs suspension under mild stirring at 4°C for 12 h to get covalent coupling between thiol-functionalized cross-linked HbNPs and polycrystalline AuE via Au-thiolated bond through dehydration process (Figure 1). The HbNPs/AuE were rinsed with 0.1 M of PB (pH 7.0) carefully and stored in PB buffer at 4°C, when not in use. The characterization of HbNPs/Au electrode was done by SEM and electrochemical impedance spectra (EIS). Below is a representation of the chemical reaction that describes the attachment of the HbNPs to the AuE.

$$\underset{\text{Polycrystalline-AuE}}{{\text{Au}}_{\text{n}}\text{-AuO }+}\underset{\text{Functionalized HbNPs}}{2(\text{HbNPs})-\text{SH}}\overset{\text{Dehvdration}}{\to }\underset{\text{Hb-E }\left(\text{Hb-electrode}\right)}{{\text{Au}}_{\text{n}}\left(\text{Au-S-HbNPs}\right)+{\text{H}}_{2}\text{O}}$$

**Figure 1:** Construction of working electrode of H2O2 biosensor Schematic representation of chemical reaction involved in the fabrication of HbNPs on AuE.

The article "An amperometric H2O2 biosensor based on hemoglobin nanoparticles immobilized on to a gold electrode" was published in 2017. Journal: Biosci Rep.

### Construction and response measurement of H_2_O_2_ biosensor

To construct the H_2_O_2_ biosensor, HbNPs/Au, as working electrode, Ag/AgCl as reference electrode, and Pt wire as counter electrode were connected through potentiostat. Cyclic voltametry (CV) of working electrode was recorded in potentiostat–galvanostat at the potential range, –0.75 to –0.25 V in 25 ml of 0.1 M sodium PB (pH 6.5) containing 0.1 ml of 100 μM H_2_O_2_. The current (in mA) was measured at different times (in s).

### Optimization of H_2_O_2_ biosensor

To optimize the working conditions of the biosensor, effects of pH, incubation temperature, time of incubation, and substrate (H_2_O_2_) concentration on biosensor response were studied. To determine the optimum pH, it was varied between 4.0 and 8.0 at an interval of 0.5 using the following buffer, each at a final concentration of 0.1 M: pH 4.0–5.0 sodium acetate buffers and pH 5.5–8 sodium PB. Similarly, to determine optimum temperature and incubation time, the reaction mixture was incubated at different temperatures (5–70°C) and time durations (1–10 s). The effect of H_2_O_2_ concentration on biosensor response was determined by varying the concentration of H_2_O_2_ in the range 1–1200 μM. The S.E.M. was calculated using the formula: S.E.M. = S.D./√*n*, where *n* is the of samples. Basically, it just tells the general variability of the points around their group means. The limit of detection (LOD) was calculated using the following formula: LOD =3σ/slope, where σ is S.D. The correlation coefficient (*R^2^*) was calculated by regression equation.

### Applications of H_2_O_2_ biosensor

Blood samples (1 ml each) were drawn from apparently healthy males and females (20 each), and persons with diagnosis of diabetes type II at Pt B.D.S. PGIMS, Rohtak Hospital and centrifuged at 2000 rpm for 10–15 min and their supernatant (serum) was collected. H_2_O_2_ content in sera was determined by the present biosensor in the similar manner as described above for its response measurement, under its optimal working conditions except that H_2_O_2_ was replaced by serum sample. The H_2_O_2_ content in serum was interpolated from standard curve between H_2_O_2_ concentrations compared with current (in mA) prepared under optimal assay conditions of biosensor (Figure 2).

The article "An amperometric H2O2 biosensor based on hemoglobin nanoparticles immobilized on to a gold electrode" was published in 2017. Journal: Biosci Rep.

**Figure 2:** Standardization of H2O2 biosensor Standard curve of H_2_O_2_ concentration by H_2_O_2_ biosensor based on HbNPs/AuE in 25-ml 0.1 M sodium PB (pH 6.5) containing 100 μM H_2_O_2_ (0.1 ml) at an applied potential of –0.25 V (compared with Ag/AgCl) with a scan rate of 20 mVs^−1^. The error bars show S.D. for *n*=3.

## Results and discussion

### Characterization of HbNPs

The average size of HbNPs as measured by TEM was between 5 and 100 nm (Figure 3a), and showed an average size of 20 nm, which enhanced the surface area of the electrode as compared with the native protein. However, this TEM image is also showing diameter of HbNPs in the higher range, i.e. 103.47–630.24 nm (average: 236.95 nm), which might be due to aggregation of HbNPs. UV and visible spectra exhibited strong absorbance peak at 280 nm, revealing a high degree of absorption of  aromatic amino acids of peptide chain confirming their NPs’ formation. The FTIR spectrum of native Hb showed distinct peaks at 1062, 1317, 1553, 1679, and 3497 cm^−1^. The strong absorption band at 1317 cm^−1^ may arise due to the stretching vibrations of C–N aromatic functional groups of protein. The medium absorption bands located at 1679 and 1553 cm^−1^ corresponds to carbonyl stretch and NH– stretch vibrations in the amide II linkage of the protein, respectively. The band at 1062 cm^−1^ indicates the presence of an amine group. In addition, there was a stretching located at 3497 cm^−1^, which could be assigned to the O H stretching vibrations, indicating the presence of hydroxyl groups. The FTIR spectrum of HbNPs showed distinct peaks at 1090, 1305, 1561, 1701, and 3488 cm^−1^ (Figure 3b). In comparison with the FTIR spectrum of the Hb and HbNPs, the major shift was observed in the carbonyl, hydroxyl, and amino groups of protein, which is due to ethanol, glutaraldehyde, and cysteamine treatment of HbNPs during their preparation.

**Figure 3:** Characterization of HbNPs. (**a**) TEM images of HbNPs. (**b**) FTIR spectra of HbNPs dispersed in 0.1 M sodium PB (pH 7.0). (**c**) SEM images of HbNPs/AuE. (**d**) EIS of bare AuE and HbNPs/AuE.

The article "An amperometric H2O2 biosensor based on hemoglobin nanoparticles immobilized on to a gold electrode" was published in 2017. Journal: Biosci Rep.

### Characterization of working electrode (HbNPs/Au) at different stages of its construction

#### By SEM

The SEM images of the surface of bare Au and HbNPs/Au are shown in Figure 3c. The stepwise modification of electrode could be seen clearly from these SEM images. The SEM image of the bare Au showed a smooth and feature-less morphology. On immobilization of HbNPs, a globular structural morphology appeared due to the interaction between HbNPs and Au, which revealed larger and effective surface area.

#### By EIS

EIS provides useful information on impedance changes on the electrode surface during the fabrication process. It was carried out to investigate immobilization of HbNPs on to Au electrode. The diameter of the semicircle at higher frequencies corresponds to the electron transfer resistance (R_CT_) which controls the electron transfer kinetics of the redox probe at the electrode interface, while the linear part at lower frequencies corresponds to Warburg diffusion process. The Nyquist plot (Figure 3d) displays EIS of HbNPs/Au in 5 mM K_3_Fe(CN)_6_/K_4_Fe(CN)_6._ The R_CT_ value for native Hb was 200 Ω which is lower than HbNPs/Au, i.e. 300 Ω. These results showed that increased R_CT_ value of HbNPs/Au electrode was due to the immobilization of HbNPs on to Au surface. This increase in R_CT_ is attributed to the fact that most of the biological molecules, including HbNPs, are poor electrical conductors at low frequencies (at least <10 kHz, applied voltage: 0.2 V) and cause hindrance to electron transfer.

### Construction and optimization of H_2_O_2_ biosensor

A novel amperometric H_2_O_2_ biosensor was developed based on covalent immobilization of HbNPs on to Au electrode. The bare AuE electrode had no oxidation and reduction peaks. The HbNPs/AuE electrode, i.e. working electrode showed optimum oxidation/reduction peak, i.e. current at a potential of –0.2 V (Figure 4), which is similar to HRP/PAN-PNMThH (–0.2 V) [31], ERGO/GCE (–0.2 V) [32] Hb/NGP (0.2 V) [20], but higher than those involving Hb/c-MWCNT (–0.365 V) [24] Hb/collagen microbelt (–0.38 V) [21], Hb/Ag sol films/GCE (–0.40 V) [22], GRCAPS/HRP/ITO (–0.45 V) [30], DNA–Hb/Au (–0.75V) [25], and lower than TTP/SPCE (–0.1V) [34], DP-AuNP/HRP/GCE (–0.05 V) [29], PtNPs/RGO/CS/Fc (–0.05 V) [28] Hb/AuNPs/L-cys/*p*-ABSA/Pt disk (0.1 V) [23], PtRu/3DGF (0.2 V) [36], Cytc/NiONPs/c-MWCNT/PANI/Au (0.28 V) [37], GPtNPs (0.45 V) [35].The biosensor showed optimum current at pH 6.5 in 0.1 M sodium PB (Figure 5a), which is similar to that of biosensor based on Cytc/NiONPs/c-MWCNT/PANI/Au [37] but lower than those involving Hb/NGP (pH 7.0) [20], Hb/collagen microbelt (pH 7.0) [21], Hb/Ag sol films/GCE (7.0) [22], Hb/AuNPs/L-cys/*p*-ABSA/Pt disk (pH 7.0) [23], Hb/collagen-MWCNT (7.0) [24], DP-AuNP/HRP/GCE (7.0) [29], GRCAPS/HRP/ITO (7.0) [30], ERGO/GCE (7.0) [32], TTP/SPCE (7.0) [34], PtRu/3DGF (7.4) [36] and higher than HRP/PAN-PNMThH (6.0) [31], TMB/HRP/PDMS/TEOS/SiO_2_NPs (5.0) [33] and DNA–Hb/Au (5.0) [25]. The optimum incubation temperature was observed at 30°C (Figure 5b), which is similar to the Cytc/NiONPs/c-MWCNT/PANI/Au (30°C) but higher than those of Hb/NGP (25°C) [20], Hb/AuNPs/L-cys/*p*-ABSA/Pt disk (25°C) [23], Hb/collagen microbelt (20°C) [21], and lower than those of PtNPs/RGO/CS/Fc (37°C) [28], GRCAPS/HRP/ITO (37°C) [30]. Figure 5c showed that there was a sharp increase in biosensor response with the increase in incubation time upto 2.5 s, after that it became constant. Hence the optimum response time of biosensor was considered as 2.5 s. The faster response time of biosensor provides the real-time analysis of the H_2_O_2_ in the serum sample. Hence, all the subsequent electrochemical experiments were carried out in 0.1 M sodium PB, pH 6.5 at 30°C. There was a linear relationship between biosensor response and H_2_O_2_ concentration in the range 1–1200 μM, the response was constant after 1200 μM (Figure 5d). The apparent *K*_m_ is an indication of protein NPs affinity. It can be calculated for immobilized protein NPs by the amperometric method, because the biosensor response is kinetic. The *K*_m_ and *V*_max_ values for the HbNPs/AuE were found to be 0.1 ± 0.01 and 5.161 ± 0.1 μA cm^−2^, respectively. The *K*_m_ value of the biosensor was lower than those of the earlier reported biosensors (45.35 μM [20] and 77.7 μM [21]). Smaller the *K*_m_ value, stronger is the affinity between HbNPs and substrate, implying that the present electrode exhibits a higher affinity for H_2_O_2_.

The article "An amperometric H2O2 biosensor based on hemoglobin nanoparticles immobilized on to a gold electrode" was published in 2017. Journal: Biosci Rep.

**Figure 4:** Response measurement of H_2_O_2_ biosensor. Cyclic voltammogram for (**A**) bare Au (**B**) HbNPs/AuE in 25-ml 0.1 M sodium PB (pH 6.5) containing 100 μM H_2_O_2_ (0.1 ml) at a scan rate of 20 mVs^−1^.

**Figure 5:** Optimization of H_2_O_2_ biosensor. (**a**) Influence of applied pH on the current response of HbNPs/AuE in 25-ml 0.1 M sodium PB (pH 6.5) containing 100 μM H_2_O_2_ (0.1 ml) at an applied potential of –0.25 V (compared with Ag/AgCl) with a scan rate of 20 mVs^−1^. The error bars show S.D. for *n*=3. (**b**) Influence of applied temperature on the current response of HbNPs/AuE in 25-ml 0.1 M sodium PB (pH 6.5) containing 100 μM H_2_O_2_ (0.1 ml) at an applied potential of –0.25 V (compared with Ag/AgCl) with scan rate of 20 mVs^−1^. The error bars show S.D. for *n*=3. (**c**) Influence of applied time on the current response of HbNPs/AuE in 25-ml 0.1 M sodium PB (pH 6.5) containing 100 μM H_2_O_2_ (0.1 ml) at an applied potential of –0.25V (compared with Ag/AgCl) with scan rate of 20 mVs^−1^. The error bars show S.D. for *n*=3. (**d**) Effect of concentration on electrochemical response of HbNPs/AuE in 25-ml 0.1 M sodium PB (pH 6.5) containing 100 μM H_2_O_2_ (0.1 ml) at an applied potential of –0.25 V (compared with Ag/AgCl) with scan rate of 20 mVs^−1^. The error bars show S.D. for *n*=3.

### Evaluation of H_2_O_2_ biosensor

There was a linear relationship between the biosensor response, i.e. current (in mA) and the H_2_O_2_ concentration in the range 1.0–1200 μM, which is better than earlier biosensors, 10–150 μM [20], 10–120 μM [25], 5–30 μM [21], 0.21–31 μM [23], 1–25 μM [22] (Supplementary Table S4). The detection limit of the present biosensor was 0.0001 μM, which is also better/lower than those of earlier biosensors: 8.24 μM [20], 0.91 μM [24], 0.4 μM [25], 0.37 μM [21], 0.1 μM [22], 0.07 μM [23]. This could be attributed to the use of NPs of Hb instead of native Hb. As the detection limit of biosensor is 0.0001 μM, it can even detect a single molecule of H_2_O_2_, showing the high sensitivity of biosensor. The average recoveries of H_2_O_2_ added in sera at levels of 0.5 and 1.0 μM were 97.77 and 98.01%, respectively (Supplementary Table S1), demonstrating the reliability of the present biosensor. The within and between batch coefficients of variation for determination of H_2_O_2_ in five sera samples on the same day and after 1 week of storage were 3.16 and 3.36%, respectively (Supplementary Table S2). These high precisions reveal the good reproducibility and consistency of the present method. The H_2_O_2_ level in sera of 20 apparently healthy subjects and persons suffering from diabetes type II, as measured by present biosensor were compared with those obtained by the standard Enzo kit method. There was a good correlation (*R^2^* =0.99) between these two methods (Figure 6a) showing the high accuracy of biosensor.

**Figure 6:** Evaluation of H_2_O_2_ biosensor. (**a**) Correlation between serum H_2_O_2_ level measured by colorimetric method (*x*-axis) and the current method (*y*-axis) employing the H_2_O_2_ biosensor based on HbNPs/AuE. (**b**) Effect of storage stability on to the activity of H_2_O_2_ biosensor.

### Interference study

The interference study was performed to assess the selectivity of the present biosensor. The HbNPs biosensor exhibited excellent anti-interference abilities with various major blood components such as citric acid, glutamic acid, uric acid, urea, and ascorbic acid at their physiological concentrations. The change in relative response in presence of citric acid, glutamic acid, uric acid, urea, and ascorbic acid was 4.20, 2.70, 1.50, 3.80, and 2.80%, respectively under the standard assay conditions. These changes (1.50–4.20%) had practically no effect on biosensor response. This practically no interference could be attributed to functioning of biosensor at lower applied potential (–0.2 V). Hence, the present biosensor could be highly selective/specific for H_2_O_2_.

The article "An amperometric H2O2 biosensor based on hemoglobin nanoparticles immobilized on to a gold electrode" was published in 2017. Journal: Biosci Rep.

### Applications of H_2_O_2_ biosensor

The H_2_O_2_ content as measured by the present biosensor was in the range from 23.9 ± 0.04 to 45.6 ± 0.05 µM (*n*=20) for sera of apparently healthy persons, which is in normal established range and from 68.2 ± 0.05 to 143 ± 0.05 µM (*n*=20) for persons suffering from diabetes type II (Supplementary Table S3).

### Storage stability of HbNPs/Au electrode

The HbNPs/Au electrode were tested every fifth day over a period of 90 days, while being stored dry at 4°C. Figure 6b shows the % of initial response of HbNPs/AuE compared with storage time. The electrode lost 10% of its initial activity after 90 days of its regular use when stored dry at 4°C. The storage stability of the present biosensor is better than earlier reported biosensors as 25 days [34], 30 days [37] which could be credited to covalent immobilization of HbNPs on to AuE.

The present biosensor could be advanced with respect to use in biomedicine or clinical settings by miniaturizing it into commercial/portable model, which could be used at the bedside of the patient. The miniaturization means designing of an electronic chip for current measuring device (potentiostat) and transformation of HbNPs/AuE into a microelectrode (like screen-printed electrode), which could be dipped into one drop of biological sample and an adopter to connect the miniaturized current device with the microelectrode. The current device needs to be battery operated and finally calibrated according to the concentration of H_2_O_2_. However, biosensor has some drawbacks such as lack of substrate specificity, requirement of expensive Au wire for construction of working electrode and cold temperature for its storage.

## Conclusion

The covalent immobilization of HbNPs on to AuE in the construction of H_2_O_2_ biosensor has resulted into its better analytical performance in terms of lower working potential (–0.2 V), which is similar to HRP/PAN-PNMThH (–0.2 V) [31], ERGO/GCE (–0.2 V) [32] Hb/NGP (0.2 V) [20], but higher than those involving Hb/c-MWCNT (–0.365 V) [24] Hb/Collagen microbelt (–0.38 V) [21], Hb/Ag sol films/GCE (–0.40 V) [22], GRCAPS/HRP/ITO (–0.45 V) [30], DNA–Hb/Au (–0.75 V) [25], and lower than TTP/SPCE (–0.1 V) [34], DP-AuNP/HRP/GCE (–0.05 V) [29], PtNPs/RGO/CS/Fc (–0.05 V) [28] Hb/AuNPs/L-cys/*p*-ABSA/Pt disk (0.1 V) [23], PtRu/3DGF (0.2 V) [36], Cytc/NiONPs/c-MWCNT/PANI/Au (0.28 V) [37], GPtNPs (0.45 V) [35], LOD (0.0001 μM) which is also better/lower than the earlier biosensors, 8.24 μM [20], 0.91 μM [24], 0.4 μM [25], 0.37 μM [21], 0.1 μM [22], 0.07 μM [23], wider linear range (1–1200 μM) which is better than earlier biosensors, 10–150 μM [20], 10–120 μM [25], 5–30 μM [21], 0.21–31 μM [23], 1–25 μM [22], rapid response (2.5 s), and higher storage stability (90 days) compared with earlier biosensors (Supplementary Table S4). Thus, covalently bound protein NPs on to AuE could be used for the construction of other improved biosensors also.

The article "An amperometric H2O2 biosensor based on hemoglobin nanoparticles immobilized on to a gold electrode" was published in 2017. Journal: Biosci Rep.

## Abbreviations

AuE: Au electrode
CS: chitosan
c-MWCNT: collagen-multiwall carbon nanotube
EIS: electrochemical impedance spectra
ERGO: electrochemically reduced graphene oxide
Fc: ferrocene
FTIR: Fourier-transform IR
FOX: 2,2 Dinitroethene-1,1-diamine
GCE: glassy carbon electrode
GPtNP: Platinum nanostructure on reduced graphene
GRCAPS: graphene capsule
GrONP: Graphene oxide nanoparticles
Hb: hemoglobin
HRP: horseradish peroxidase
ITO: indium tin oxide
LOD: limit of detection
L-cys: L-Cysteine
NGP: nanographene platelet
NiONP: nickel oxide nanaoparticle
NP: nanoparticle
PANI: polyalinine
PAN-PNMThH: poly(aniline-co-N-methyllanthionine)
PB: phosphate buffer
PDMS: polydimethylsiloxane
PtRu: Platinum-Ruthenium bimetallic catalyst
*p*-ABSA: *p*-aminobenzene sulphonic acid
p123: Pluronic P-123
R_CT_: electron transfer resistance
RGO: reduced graphene oxide
PGE: Pencil graphite electrode
ROS: reactive oxygen species
*R^2^*: correlation coefficient
SPCE: Screen printed carbon electrode
TEOS: tetraethylorthosilicate
TMB: 3,3′,5,5′-teramethylbencidine
TTP: turnip tissue paper
3DGF: Three dimensional graphene foam
